# Effect of Ambient Lights on the Accuracy of a 3-Dimensional Optical Scanner for Face Scans: An In Vitro Study

**DOI:** 10.1155/2022/2637078

**Published:** 2022-08-05

**Authors:** Punrit Thongma-Eng, Pokpong Amornvit, Patcharawan Silthampitag, Dinesh Rokaya, Attavit Pisitanusorn

**Affiliations:** ^1^Department of Prosthodontics, Faculty of Dentistry, Chiang Mai University, Chiang Mai 50200, Thailand; ^2^PPFACEDESIGN, The S Clinic, Bangkok 10120, Thailand; ^3^Department of Clinical Dentistry, Walailak University International College of Dentistry, Walailak University, Bangkok 10400, Thailand

## Abstract

Most 3D scanners use optical technology that is impacted by lighting conditions, especially in triangulation with structured-light or laser techniques. However, the effect of ambient lights on the accuracy of the face scans remains unclear. The purpose of this study is to investigate the effect of ambient lights on the accuracy of the face scans obtained from the face scanner (EinScan Pro 2X Plus, Shining 3D Tech. Co., LTD., Hangzhou, China). A head model was designed in Rhinoceros 5 software (Rhino, Robert McNeel and Associates for Windows, Washington DC, USA) and printed with 200 micron resolution of polylactic acid and was dented with 2.0 mm of carbide bur to aid in superimposition in software. The head model was measured by a coordinate-measuring machine (CMM) to generate a reference stereolithography (STL) file as a control. The face model was scanned four times under nine light conditions: cool white (CW), warm white (WW), daylight (DL), natural light (NL), and illuminant (9w, 18w, 22w). Scan data were exported into an STL file. The scan STL files obtained were compared with the reference STL file by 3D inspection software (Geomagic Control X version 17, Geomagic, Morrisville, NC, USA). The deviations and root mean square errors (RMSEs) between the reference model (trueness) and within the group (precision) were selected for the statistical analysis. The statistical analysis was done using SPSS 20.0 (IBM Company, Chicago, USA). The trueness and precision were evaluated with the one-way ANOVA with multiple comparisons using the Tukey method. For trueness, the scanner showed the lowest RMSE under the NL group (77.18 ± 3.22) and the highest RMSE under the 18w-DL group (95.33 ± 6.89). There was a statistically significant difference between the NL group and the 18w-DL group (*p* < 0.05) for trueness. Similarly, for precision, the scanner showed the lowest RMSE under the NL group (56.92 ± 4.56) and the highest RMSE under the 9w-CW group (78.52 ± 10.61). There was statistically significant difference between NL, 18w-WW, 18w-CW, 18w-DL, 22w-WW, 22w-DL, 9w-CW, 9w-WW, and 9w-DL (*p* < 0.05) for the precision. Ambient lights affected the face scans. Under the natural light condition, the face scanner had the best accuracy in terms of both trueness and precision. The 18w-DL and 9w-WW conditions showed the least trueness whereasthe 9w-CW and 9w-DL conditions showed the least precision.

## 1. Introduction

Traditionally, in plastic surgery and dentistry, patients' faces were analyzed from photographs of the patients taken from various angles. However, with the advancements of digital technologies including optical scanning technologies, face analysis can be done using two-dimensional (2D) and three-dimensional (3D) technologies [1–4]. Today, 3D facial models can be obtained from 3D scanners and these have been incorporated in clinical dentistry and medicine such as in orthodontics, orthognathic surgery, plastic surgery, prosthodontics, and so on for preoperative diagnosis, evaluation, and postoperative outcome simulation [5–7].

Various 3D facial scanning technologies are used in clinical dentistry, such as photogrammetry, stereophotogrammetry, structured-light scanning, and laser scanning [4, 8]. Photogrammetry and stereophotogrammetry are photo-based techniques that use a series of photographs of patients from different angles to generate facial reconstruction through 3D software, while laser and structured-light scanning obtained facial reconstruction through a triangulation technique, projected light patterns onto external surfaces, and captured distortion of the pattern by a high-resolution camera [8–10].

In the last 20 years, there has been growing interest in 3D scanning technologies in medicine and dentistry. Fourie et al. [11] reported that laser scanning, CBCT, and stereophotogrammetry were acceptable for use in the clinic. Similarly, Ghoddousi et al. [12] reported that the stereophotogrammetry technique and 2D photographs compared with direct measurement were reliable and clinically accepted. In the meantime, the advent of 3D technology not only makes 3D reconstruction feasible but also more accurate for scanning. Beaumont et al. [13], Zhao et al. [14], and Gomes et al. [15] also reported that accurate measurements can be acquired by these systems (infrared, structured-light, laser, and stereophotogrammetry). The latest systematic review in 2018 [16] reported that all studies disclosed a deviation close to 1.0 mm.

All 3D scanners that use optical technology are impacted by lighting conditions, especially in structure-light or laser techniques [17]. The ambient light can decrease the intensity of light projected from the scanners. Thus, the reconstruction quality by point clouds will be degraded. Voisin et al. [18] reported that the accuracy of scans were affected not only by the ambient light but also the colour. Gupta et al. [19] also recommended decreasing the illuminance of ambient light or increasing the intensity of projected light to maintain scanning accuracy. Additionally, researchers reported that ambient light affects the measure coordinated in 3D scanning and mentioned that it is most appropriate for digitization in the absence of ambient lights [20].

The “accuracy” includes both trueness and precision [21]. The trueness is the capacity of the scanner to produce 3D construction as close to its true dimension as possible, while precision is the capacity of the scanner to produce 3D construction within the acquired parameters by repeated scanning under the same conditions.

It is important to study the effect of ambient light on the accuracy of facial scans. Hence, this study aimed to study the effect of the ambient lights on the accuracy of the specific face scans. Also, the accuracy of the scans was measured under various light conditions.

## 2. Materials and Methods

The study includes scanning the face of the head model under various ambient lights and a comparison of the accuracy of the specific face scans.  Figure 1 shows the overview of this study.

### 2.1. Head Model Acquisition

A head model was designed in Rhinoceros 5 software (Rhino, Robert McNeel and Associates for Windows, Washington DC, USA) with the shape and size close to human face (anonymous) as shown in Figure 2. Then, the face model was printed with polylactic acid polymer by the fused deposition modeling technique (FDM) with 200 micron resolution [22]. Grey-colored nylon was chosen because of the properties of light capturing and the texture similar to normal human skin. Then, three points were demarked with 2.0 mm in diameter of carbide bur on the face model in different spatial planes (nasion, right chelion, and left chelion) to aid in the future superimposition of the 3D model in software. The face model was measured by a coordinating measuring machine (CMM) (Global S, Hexagon Manufacturing Intelligence World Headquarter office, Surrey, Great Britain) at 25 micron resolution to generate a reference stereolithography (STL) file.

### 2.2. Face Model Scanning

Scanners operated in handheld quick scan mode following the technical specifications combined with texture scan mode provides an accuracy of 0.1 mm. Ambient light settings are shown in Figures 3 and 4. Settings were divided into 9 groups: (1) 9w-WW, (2) 9w-CW, (3) 9w-DL, (4) 18w-WW, (5) 18w-CW, (6) 18w-DL (7), 22w-WW, (8) 22w-DL (EveLighting Co., LTD., Bangkok, Thailand), and (9) natural light; a room with window, switched off all ceiling lights, 500 lux light through lux meter (Digital lux meter, Jedto LS-1010BS, Protronics Co., LTD., Pathum Thani, Thailand) [23]. Groups 1–8 were scanned in a dark room to eliminate external light. Other confounding factors controlled by the operator were the distance between the rotation axis of the head model and the scanner, and the scanning technique. Then, the four scans for each group were done using an infinite population standard deviation (*σ*) = 5, error (d) = 5, and alpha (*α* = 0.05) as shown in the following equation:

(1) $$\begin{array}{c} \text{mean}=\frac{z_{1-\left(\alpha /2\right)}^{2}\sigma^{2}}{d^{2}}, \end{array}$$

where *σ* = standard deviation, *d* = error, and *α* = alpha.

### 2.3. Comparison

The scanned data were analyzed using the 3D inspection software (Geomagic Control X version 17, Geomagic, Morrisville, NC, USA). The scanned data were aligned to the reference data by using Local Based on Picked point from software. Then, the deviations and root means square errors (RMSE) were selected for statistical analysis between the reference model (trueness) and within the group (precision). The trueness and precision were evaluated with the One-way ANOVA with multiple comparisons using the Tukey method. The significance level was chosen at *p* < 0.05.

## 3. Results

For trueness, the results are shown in Table 1 and Figure 5. The mean deviations of RMSE were 91.25 ± 4.93 for 9w-WW, 91.25 ± 10.56 for 9w-CW, 92.45 ± 9.39 for 9w-DL, 91.78 ± 5.36 for 18w-WW, 88.73 ± 4.73 for 18w-CW, 95.33 ± 6.89 for the 18w-DL, 82.95 ± 2.78 for 22w-WW, 83.40 ± 7.30 for 22w-DL, and 77.18 ± 3.22 for NL. The scanner had the lowest RMSE under the NL group and the highest RMSE under the 18w-DL group. It showed that there was a statistically significant difference between the NL group and the 18w-DL group (*p* < 0.05).

For the precision, the results are shown in Table 2 and Figure 6. The mean deviations of RMSE are 72.38 b ± 7.22 for 9w-WW, 78.52 ± 10.61 for 9w-CW, 73.84 ± 12.96 for 9w-DL, 70.67 ± 9.66 for 18w-WW, 62.28 ± 3.18 for 18w-CW, 70.70 ± 10.63 for 18w-DL, 62.10 ± 2.69 for 22w-WW, 65.30 ± 4.41 for 22w-DL, and 56.92 ± 4.56 for NL as shown in Table 2 and Figure 5. The scanner had the lowest RMSE in the NL group and the highest RMSE in the 9w-CW group. It showed that there was statistically significant difference between NL, 18w-WW, 18w-CW, 18w-DL, 22w-WW, 22w-DL, 9w-CW, 9w-WW, and 9w-DL (*p* < 0.05).

For the light power (Watt), there is no significant difference among the groups in the same ambient light group.

## 4. Discussion

This study investigated the impact of ambient lights on the accuracy of the face scans, and we found that the ambient lights affect the accuracy of the face scans.

This study found that the scanner had the best accuracy (the lowest RMSE in both trueness and precision) under natural light conditions (NL group) which represented the optimal time at around noon. The scanner had the least accuracy under the 18w-DL group for trueness and 9w conditions for precision as shown in Figure 7. Normally, most dental clinics use 18w or more LED lamps and daylight temperature in their settings. Therefore, some scan data could not be captured or the captured data were represented incorrectly. Thus, errors can occur in these situations.

In this investigation, the software showed that the range of discrepancies between the measured data and the referenced data was less than 0.5 mm in all groups. According to a previous study [22], EinScan Pro 2X plus had shown no significant difference in the *X* and *Y* axis except for the *Z* axis. While the lay perception was 1.83 mm as the minimum threshold for midline discrepancy. Therefore, all groups were clinically acceptable at discrepancy up to 2.0 mm. It was suitable to use in tasks with an accuracy greater than 2.0 mm [24, 25].

In this study, the methodology was designed to minimize the influence of other factors on the accuracy by using the same operators, the distance between the rotational axis of the object and scanner, scan strategy, and calibration of the scanner before scanning. Additionally, EinScan Pro 2X Plus has shown the best accuracy among other scanners for face scanning in the previous study [22]. Furthermore, most previous studies [23, 26, 27] applied the best-fit algorithm to their dataset. The best-fit algorithm uses the signed nearest neighbor method to find the deviation. Where the reference data were not superimposed exactly at the same position as every measured dataset, these become a confounding factor in their investigation. Larger data and more differences in data result in more errors during superimposition [28]. Hence, in this study, we used three markers with Local Based of Picked Point instead of the best-fit algorithm.

Regarding the limitation of our study, we used a model to study the influence of ambient lights but not in real patients. Human skin is composed of melanin, vessels, and an oily surface. Layered and other optic properties such as absorption and scattering affected the optic scanner differently. Thus, this study used material that had a refractive index in the range of human skin (refractive index of normal human skin ranges from 1.41–1.49 [29]). To eliminate the movement while scanning and other properties of human skin, this model was chosen instead of a human subject. In the clinic, the accuracy of face scans can be affected by various factors such as the refractive index, scan strategies, and software version. Moreover, we selected only one 3D scanner in this study. Further investigations can be done using various scanners in the real clinical setting. But this study will form a guide for future clinical studies.

## 5. Conclusions

The following conclusions can be drawn:

1. The ambient lights influence the accuracy (trueness and precision) of the face scans.
2. Under natural light conditions, EinScan Pro 2X Plus had the best accuracy in terms of both trueness and precision. In contrast, under 18w-DL and 9w conditions, the scanner had the least accuracy of trueness and precision, respectively. We recommend that face scanning should be performed under natural light conditions for the best accuracy.

## Figures and Tables

**Figure 1:** Overview of the study. CMM = coordinate-measuring machine.

**Figure 2:** Head model and close-up image of marker.

**Figure 3:** Equipment setting (top view).

**Figure 4:** Equipment setting (lateral view).

**Figure 5:** Results of trueness: bar chart with error bars for standard deviation (w = Watts, WW = warm white, CW = cool white, DL = daylight, and NL = natural light).

**Figure 6:** Results of precision: bar chart with error bars for standard deviation (w = Watts, WW = warm white, CW = cool white, DL = daylight, and NL = natural light).

**Figure 7:** . The color-coded map showing 3D comparison of all groups: (a) 9w-WW, (b) 9w-CW, (c) 9w-DL, (d) 18w-WW, (e) 18w-CW, (f) 18w-DL, (g) 22w-WW, (h) 22w-DL, and (i) NL.

**Table 1:** Root mean square error (RMSE, *µ*m) for trueness.

Ambient light		9w			18w			22w		NL
		WW	CW	DL	WW	CW	DL	WW	DL	
Trueness	Mean	91.25	91.25	92.45	91.78	88.73	95.33^*∗*^	82.95	83.40	77.18^*∗*^
	SD	4.93	10.56	9.39	5.36	4.73	6.89	2.78	7.30	3.22

^∗^Statistically significant at *p* < 0.05. w = Watts, WW = warm white, CW = cool white, DL = daylight, and NL = natural light.

**Table 2:** Root mean square error (RMSE, *µ*m) for precision.

Ambient light		9w			18w			22w		NL
		WW	CW	DL	WW	CW	DL	WW	DL	
Precision	Mean	72.38^*∗*^	78.52^*∗*^	73.84^*∗*^	70.67^*∗*^	62.28^*∗*^	70.70^*∗*^	62.10^*∗*^	65.30^*∗*^	56.92^*∗*^
	SD	7.22	10.61	12.96	9.66	3.18	10.63	2.69	4.41	4.56

^∗^Statistically significant at *p* < 0.05. w = Watts, WW = warm white, CW = cool white, DL = daylight, and NL = natural light.

## Data Availability

The data used to support the findings of this study are available from the corresponding author upon reasonable request.

## References

[1] Berssenbrügge P., Berlin N. F., Kebeck G. (2014). 2D and 3D analysis methods of facial asymmetry in comparison. *Journal of Cranio-Maxillofacial Surgery*.

[2] Humagain M., Rokaya D. (2019). Integrating digital technologies in dentistry to enhance the clinical success. *Kathmandu University Medical Journal*.

[3] He M. (2021). Research on face image digital processing and recognition based on data dimensionality reduction algorithm. *Computational Intelligence and Neuroscience*.

[4] Amornvit P., Rokaya D., Peampring C., Sanohkan S. (2020). Confocal 3D optical intraoral scanners and comparison of image capturing accuracy. *Computers, Materials & Continua*.

[5] Liu Y. S., Ye H. Q., Gu M. (2014). Application of patient-participated digital design in esthetic rehabilitation of anterior teeth. *Beijing da xue xue bao. Yi xue ban= Journal of Peking University. Health Sciences*.

[6] Wei Y., Chen G., Han B., Hu X., Zhang H., Deng X. (2014). Three-dimensional imaging for quantitative evaluation of facial profile of edentulous patients before and after complete dentures restoration. *Beijing da xue xue bao*.

[7] Amornvit P., Rokaya D., Sanohkan S. (2021). Comparison of accuracy of current ten intraoral scanners. *BioMed Research International*.

[8] Ye H., Lv L., Liu Y., Zhou Y. (2016). Evaluation of the accuracy, reliability, and reproducibility of two different 3D face-scanning systems. *International Journal of Prosthodontics*.

[9] Ma L., Xu T., Lin J. (2009). Validation of a three-dimensional facial scanning system based on structured light techniques. *Computer Methods and Programs in Biomedicine*.

[10] Petrides G., Clark J. R., Low H., Lovell N., Eviston T. J. (2020). Three-dimensional scanners for soft tissue facial assessment in clinical practice. *Journal of Plastic Reconstructive & Aesthetic Surgery*.

[11] Fourie Z., Damstra J., Gerrits P. O., Ren Y. (2011). Evaluation of anthropometric accuracy and reliability using different three-dimensional scanning systems. *Forensic Science International*.

[12] Ghoddousi H., Edler R., Haers P., Greenhill D. (2007). Comparison of three methods of facial measurement. *International Journal of Oral and Maxillofacial Surgery*.

[13] Beaumont C. A., Knoops P. G., Borghi A. (2017). Three-dimensional surface scanners compared with standard anthropometric measurements for head shape. *Journal of Cranio-Maxillofacial Surgery*.

[14] Zhao Y. J., Xiong Y. X., Yang H. F., Wang Y. (2014). Evaluation of measurement accuracy of three facial scanners based on different scanning principles. *Beijing da xue xue bao. Yi xue ban= Journal of Peking University. Health Sciences*.

[15] Gomes C. F. D., Libdy M. R., Normando D. (2019). Scan time, reliability and accuracy of craniofacial measurements using a 3D light scanner. *Journal of oral biology and craniofacial research*.

[16] Bohner L., Gamba D. D., Hanisch M. (2019). Accuracy of digital technologies for the scanning of facial, skeletal, and intraoral tissues: a systematic review. *The Journal of Prosthetic Dentistry*.

[17] Lemeš S., Zaimović-Uzunović N. Study of ambient light influence on laser 3D scanning.

[18] Voisin S., Foufou S., Truchetet F., Page D. L., Abidi M. A. (2007). Study of ambient light influence for three-dimensional scanners based on structured light. *Optical Engineering*.

[19] Gupta M., Yin Q., Nayar S. K. Structured light in sunlight.

[20] Blanco D., Fernandez P., Cuesta E., Suarez C. Influence of ambient light on the quality of laser digitized surfaces.

[21] Accuracy ISO (1994). *(Trueness and Precision) of Measurement Methods and Results-Part 1: General Principles and Definitions*.

[22] Amornvit P., Sanohkan S. (2019). The accuracy of digital face scans obtained from 3D scanners: an in vitro study. *International Journal of Environmental Research and Public Health*.

[23] Revilla-León M., Jiang P., Sadeghpour M. (2020). Intraoral digital scans-Part 1: influence of ambient scanning light conditions on the accuracy (trueness and precision) of different intraoral scanners. *The Journal of Prosthetic Dentistry*.

[24] Parrini S., Rossini G., Castroflorio T., Fortini A., Deregibus A., Debernardi C. (2016). Laypeople’s perceptions of frontal smile esthetics: a systematic review. *American Journal of Orthodontics and Dentofacial Orthopedics*.

[25] Knoops P. G., Beaumont C. A., Borghi A. (2017). Comparison of three-dimensional scanner systems for craniomaxillofacial imaging. *Journal of Plastic, Reconstructive & Aesthetic Surgery*.

[26] Arakida T., Kanazawa M., Iwaki M., Suzuki T., Minakuchi S. (2018). Evaluating the influence of ambient light on scanning trueness, precision, and time of intra oral scanner. *Journal of prosthodontic research*.

[27] Revilla-Leon M., Subramanian S. G., Krishnamurthy M., aman V. (2020). Clinical study of the influence of ambient light scanning conditions on the accuracy (trueness and precision) of an intraoral scanner. *Journal of Prosthodontics*.

[28] Güth J.-F., Edelhoff D., Schweiger J., Keul C. (2016). A new method for the evaluation of the accuracy of full-arch digital impressions in vitro. *Clinical Oral Investigations*.

[29] Lister T., Wright P. A., Chappell P. H. (2012). Optical properties of human skin. *Journal of Biomedical Optics*.

